The article "Seed priming with growth regulators modulates production, physiology and antioxidant defense of Indian squash (Praecitrullus fistulosus) under semi-arid conditions" was retracted in 2022. Reasons: compromised peer review; a conflict of interest; concerns about the authorship.

# Seed priming with growth regulators modulates production, physiology and antioxidant defense of Indian squash (*Praecitrullus fistulosus*) under semi-arid conditions

**DOI:** 10.1371/journal.pone.0265694

**Published:** 2022-04-14

**Authors:** Rafi Qamar, Sanaullah Khan, Muhammad Ehsan Safdar, Atique-ur-Rehman, Abdul Rehman, Hafiz Muhammad Rashad Javeed, Muhammad Ather Nadeem, Rashid Al-Yahyai, Jawaher Alkahtani

**Affiliations:** 1 Department of Agronomy, College of Agriculture, University of Sargodha, Sargodha, Pakistan; 2 Department of Agronomy, Bahauddin Zakariya University, Multan, Pakistan; 3 Department of Environmental Sciences, COMSATS University Islamabad, Vehari Campus, Pakistan; 4 Department of Plant Sciences, College of Agricultural and Marine Sciences, Sultan Qaboos University, Muscat, Oman; 5 Department of Crop Science, University of Reading, Reading, United Kingdom; 6 Department of Botany and Microbiology, College of Science, King Saud University, Riyadh, Saudi Arabia; Ghazi University, PAKISTAN

## Abstract

Indian squash (*Praecitrullus fistulosus*) crop faces heat and drought during its growth that is considered the most important abiotic stress in semi-arid areas. Seed priming with growth regulators enhances stress tolerance; hence, mitigates the adverse effects of unpredictable stresses due to adverse weather conditions. This two-year (2019 and 2020) study was conducted to infer the role of seed priming in improving heat tolerance of Indian squash (cultivar Sahavi) through improvement in physiological and antioxidant defense systems. Six treatments that included no priming (control), hydropriming, priming with indole acetic acid (IAA) at 100 mg L^-1^, salicylic acid (SA) at 50 mg L^-1^, ascorbic acid (AA) at 100 mg L^-1^ and thiourea at 500 mg L^-1^ each for 06 hours) were included in the study. Results revealed that priming with AA and SA significantly (*P* ≤ 0.05) enhanced germination (39 and 47%), germination index (57 and 58%), plant height (23 and 22%), vine length (15 and 14%), number of fruits per plant (62%), fruit weight per plant (66 and 67%), economic yield (32%), photosynthesis rate (18 and 17%), protein content (10%), proline (23%), glycine betaine (3%), malondialdehyde content (11 and 10%) and catalase activity (24%) compared to control treatment. Furthermore, seed priming with AA and SA significantly (*P* ≤ 0.05) shortened the mean germination time (25 and 28%) compared to the control. The results indicated that AA and SA had significant potential to mitigate adverse effects of heat stress in Indian squash. Findings from this study showed that seed priming with AA and SA promoted heat-stress tolerance and enhanced growth and productivity of Indian squash.

The article "Seed priming with growth regulators modulates production, physiology and antioxidant defense of Indian squash (Praecitrullus fistulosus) under semi-arid conditions" was retracted in 2022. Reasons: compromised peer review; a conflict of interest; concerns about the authorship.

## Introduction

Indian squash (*Praecitrullus fistulosus*) locally known as *tinda* or *dilpasand* is cooked as a vegetable in Pakistan. It is a rich source of vitamins A, B and C. It belongs to *Cucurbitaceae* family and cultivated during *Zaid Rabi* (February to end of April) and *Kharif* season (mid-June to end of July). Therefore, it is available in the market from May to November. It is a very sensitive crop and can’t tolerate low temperatures [1]. It requires 30 to 35 °C temperature during daytime and 18 °C or below at nighttime for development and fruit formation. However, the optimum temperature is 25 °C for its better growth and production [1]. In Pakistan, Indian squash is cultivated on 5.86 thousand hectares which produced 57.67 thousand tones with an average production of 9839 kg per hectare [2]. *Kharif* season production is lower than *Zaid rabi* season due to high temperature (40 to 45 °C) which significantly reduces its production due to oxidative stress that leads to restriction in normal functioning and physiology [3]. During high-temperature stress, the plant produces and accumulates osmoprotectants such as proline and glycine betaine as an adaptation mechanism [4]. Therefore, the major cause of its lower yield during *Kharif* season is high temperature and scanty rainfall which leads to poor crop establishment at farmer’s fields. Different techniques may be applied to overcome the destructive effects of the environment, including mulching, sprinkler irrigation, and seed priming.

Seed priming may improve plant emergence and development that leads to higher production [5]. Different chemicals like plant hormones and antioxidants are applied to protect cell death at apical meristem, especially DNA damage [6] to ensure higher germination and plant development during environmental extremes [7]. Moreover, seed priming enhances seed germination under harsh weather conditions through shortening time to 50% emergence, and average time to germination [8]. Seed priming activates metabolic processes that are essential for germination process and leads to consistency in germination; therefore, considerably improves crop production [9]. Seed priming brings significant improvements in enzymes’ activities which are directly involved in the metabolism of stored food in seed [10]. Furthermore, seedlings grown from primed seeds have a higher antioxidative defense that triggers stress inhibiting and late embryogenesis proteins [11].

Recently, hydropriming technique has been applied to overcome the adverse effects of abiotic stresses. However, hydro-priming doesn’t show fruitful results under abrupt environmental changes as compared to priming with growth regulators. Mitigation of harmful effects of climate change on crop production can be possible through the application of plant growth regulators (PGRs) [12]. Recently, it has been proved that PGRs act as signaling molecules that improve different physiological processes [13], including enzyme performance [14], photosynthesis rate [15] and plant development [16]. Moreover, these reduce the detrimental effects of environmental fluctuation through the modification of the internal physiological processes of plants [17].

The article "Seed priming with growth regulators modulates production, physiology and antioxidant defense of Indian squash (Praecitrullus fistulosus) under semi-arid conditions" was retracted in 2022. Reasons: compromised peer review; a conflict of interest; concerns about the authorship.

Among growth regulators, indole acetic acid (IAA) improves seedling growth and development by targeting the plant growing sites and stimulates seed germination, cell growth and elongation, root initiation and cell growth at the apex of shoot [18–20]. Ascorbic acid (AA) is another growth regulator that performs various critical functions and acts as a leading cofactor in various essential physiological functions and development of antioxidant enzymes [21]. External application of AA is advisable under high temperature (44 °C) [22] which effectively improves germination and growth attributes [23] through improvement in antioxidant enzymes activities [24]. Similarly, salicylic acid (SA) is recognized as an endogenic plant regulator, which is involved in many physiological and biochemical developments of plants under varying temperatures [25]. Several studies have indicated that SA application through seed priming improved germination and growth [23] of various crops through developing tolerance against high temperatures [26]. Thiourea is a synthetic growth regulator consisting of nitrogen and sulfur. The application of thiourea modulates various physiological events such as photosynthetic rate, proline content, antioxidant enzyme system and osmotic adjustment during plant development under higher temperatures [27]. Seed priming with thiourea resulted in significantly improved crop production under high temperatures, i.e., 35 °C and 45 °C by stimulating enzymes and nutrient availability [28].

There is no study conducted indicating the role of seed priming with PGRs in enhancing Indian squash yield under high temperatures as experienced in field conditions. It was hypothesized that seed priming of *kharif*-sown Indian squash with PGRs under field conditions will mitigate the adverse impacts of heat stress and result in better yield. For this purpose, IAA, SA, AA and thiourea were utilized to investigate their role in enhancing Indian squash production under field conditions in semi-arid climatic conditions.

## Materials and methods

### Experiment site and soil

The current study was performed at Agronomic Research Area, College of Agriculture, University of Sargodha, Punjab, Pakistan, during *Kharif* seasons of 2019 and 2020. The experimental site is located at 32.08 °N, 72.67 °E at an altitude of 193 m. The climate of Sargodha region is semi-arid having yearly precipitation of 400±5 mm. About 70% or more precipitation fall in July and September (Source: Agro-Metrological Lab, University of Sargodha). Summary of the environmental conditions during the entire growing period of 2019 and 2020 is shown in Fig 1. For physico-chemical analysis, the soil was oven-dried, ground and passed through a 2 mm sieve before the start of the experiment during 2019 and 2020. The physico-chemical properties of the soil are given in Table 1. The soil used in this study belongs to Hafizabad series having a sandy loam texture [29].

The article "Seed priming with growth regulators modulates production, physiology and antioxidant defense of Indian squash (Praecitrullus fistulosus) under semi-arid conditions" was retracted in 2022. Reasons: compromised peer review; a conflict of interest; concerns about the authorship.

**Fig 1:** Meteorological data recorded at College of Agriculture, University of Sargodha, Sargodha, Punjab, Pakistan during 2019 and 2020.

**Table 1:** Physio-chemical characteristics of the experimental site at College of Agriculture, University of Sargodha, Sargodha, Pakistan.

Soil properties	Values		Analytical method
	2019	2020	
Mechanical composition			Bouycous hydrometer method [30]
Sand (g kg^-1^)	469 ± 2.5	469 ± 2.5	
Silt (g kg^-1^)	238 ± 2.1	238 ± 2.1	
Clay (g kg^-1^)	288 ± 1.4	288 ± 1.4	
Textural class	Sandy Loam		
Chemical composition			
Saturation percentage	40.17 ± 1.18	40.71 ± 1.13	US Salinity Laboratory Staff
pH	7.5 ± 0.03	7.6 ± 0.03	Beckman’s Glass electrode pH meter [31]
ECe (μS cm^-1^)	15.40 ± 22.1	16.80 ± 28.74	Conductivity bridge from 1:2:5 soil water ratio
Organic content (g kg^-1^)	7.43 ± 0.60	7.39 ± 0.30	Walkley and Black method [30]
Total soil N (mg kg^-1^)	4.08 ± 8.15	4.12 ± 7.30	Modified Kjeldahl method [30]
NaHCO_3_ Extractable-P (mg kg^-1^ soil)	7.41 ± 0.10	7.72 ± 0.30	Olsen’s method [31]
Available potassium (mg kg^-1^)	269 ± 12.10	271 ± 11.12	Flame photometric [31]

Given values are the average of three replication followed by (±) standard error.

### Seed priming treatments

Seeds of Indian Squash cultivar Sahavi were obtained from the Vegetable Section, Ayub Agricultural Research Institute, Faisalabad, Pakistan. The seeds were surface sterilized with 1% sodium hypochlorite before seed priming. After five minutes, seeds were washed three times with distilled water to completely remove residues. Then seeds were air-dried and treated with respective seed priming agent, i.e., PGRs. The seeds were primed with indole acetic acid (IAA) at 100 mg L^-1^, salicylic acid (SA) at 50 mg L^-1^, ascorbic acid (AA) at 100 mg L^-1^, thiourea at 500 mg L^-1^, and distilled water (hydropriming). An untreated control was also kept for comparison. The concentrations were determined based on earlier studies [23]. The seeds were dipped in the aerated solutions of PGRs for 24 hours and then dried to their original weight under shade.

The article "Seed priming with growth regulators modulates production, physiology and antioxidant defense of Indian squash (Praecitrullus fistulosus) under semi-arid conditions" was retracted in 2022. Reasons: compromised peer review; a conflict of interest; concerns about the authorship.

### Crop sowing and management

Experimental field was irrigated and plowed twice with moldboard plow followed by two planking for soil preparation during both years. Seedbed was prepared with the help of a bed shaper and the bed size was kept 4.5 m × 3 m. The experiment was laid out in randomized complete block design with three replications. The seeds were sown manually by employing *Choppa* method using 1.7 kg seed ha^-1^. Seed moisture content was 5.32% measured on a dry weight basis. The planting distance was 1.5 m between rows and 0.9 m within rows. Three seeds per hill were sown at a depth of 2 cm. The seedlings were thinned to one per hill at 3^rd^ week after sowing when 2 to 3 true leaves emerged. First irrigation was applied after 3 days of sowing, while succeeding irrigations were applied 2 times per week. The plant available water contents were maintained at 70% of the field capacity due to coarse-textured soil. For this purpose, Tensiometer (Model RM 627) was used to optimize irrigation. The crop was fertilized with 120:80:50 kg nitrogen:phosphorus:potash ha^-1^ at the time of sowing in which whole of the phosphorus and potash, while one-third of the nitrogen were incorporated. The remaining nitrogen was fertilized in two doses, 1^st^ at shoot elongation and 2^nd^ at flowering stage. Manual weeding was done at 3^rd^, 5^th^ and 7^th^ weeks after sowing to control the weeds. Polo at 150 ml/lit + Trichlorophone 80 SP at 1680 g/ha were sprayed to control the insect pests. For the control of diseases, carbamate fungicide was used. The fruits were detached manually at maturity to record economic yield. All the necessary inputs, and pest management operations were implemented across the growing seasons uniformly based on the crop requirements.

### Data collection

Seedling emergence, growth, yield, physiological traits, and antioxidant enzymes were determined during and after the harvest of the crop. Seedling emergence percentage (EP) was calculated by adopting the procedure of Association of Official Seed Analysts [32]

$$EP=\frac{Emerged\;seeds\;}{Total\;seeds}\;\times 100$$

The emergence index (EI) was worked out by applying the formula given by Association of Official Seed Analysts [32]

$$EI=\frac{No.\;of\;emerged\;seeds}{Days\;of\;first\;count}+\frac{No.\;of\;emerged\;seeds}{Days\;of\;final\;count}$$

Mean emergence time (MET) was computed according to the formula of Ellis and Roberts [33]:

MET=∑(Dn)∑n

Here, *n* shows germinated seed, *D* shows the number of days.

The article "Seed priming with growth regulators modulates production, physiology and antioxidant defense of Indian squash (Praecitrullus fistulosus) under semi-arid conditions" was retracted in 2022. Reasons: compromised peer review; a conflict of interest; concerns about the authorship.

Vine length was recorded by measuring the length of five randomly selected plants from each experimental unit with the help of measuring tape. The number of fruits per plant was noted by averaging the number of fruits harvested from five randomly tagged plants. For fruit weight, ten fruits were selected from the above-tagged plants and weighed using electrical balance (Model Number: HC2204) and averaged. Economic yield (Mg/ha) was recorded by weighing 1^st^, 2^nd^, and 3^rd^ pickings from randomly marked five plants and then all fruit harvest data were cumulated, averaged, and converted into Mg/ha.

On the 60^th^ day, five leaves from each experimental unit were randomly picked and put in a chamber of an Infrared Gas Analyzer (IRGA) one by one. The photosynthesis rate was recorded from 11.00 to 12.00 am. During readings IRGA chamber was set according to guidelines of Zekri [34] and Moya et al. [35]. The chamber was set at 403.3 mmol m^-2^ s^-1^ molar flow rate, 99.90 KPa atmospheric pressure, 6.0 to 8.9 mbar vapor pressure, 1711 μmol m^-2^ s^-1^ photosynthetically active radiation, 28.40 to 32.40 °C leaf temperature, 22.40 to 27.90 °C ambient temperature, and 352 μmol mol^-1^ ambient CO_2_ concentration. The k-leaves were blended into a medium of pH 7.0 having a buffer solution of 50 mM potassium phosphate for measuring protein contents [36]. To determine the protein in the sample, 5 μL of liquid and 0.1 N NaCl were added into 1.0 mL Bradford dye. The whole solution was kept for 5 minutes for the formation of a protein-dye complex. Then a spectrophotometer was used to record absorbance at 595 nm. Proline was estimated by following the protocol of Bates et al. [37]. For this purpose, 200 mg leaf samples were homogenously mixed in 12 mL 3% aqueous H_2_SO_4_. Then 2 mL of the above filtrate was added for reaction in 2 mL of acid ninhydrin plus 2 mL acetic acid at 100 °C, and the chemical reaction was terminated after 1 hour. The compound was added into a 4 mL solvent and homogenized smartly for 10 to 15 sec. The colored chemical having solvent was extracted in liquid form and warmed at room temperature. Solvent reading was registered at 520 nm as a blank value. Proline content (mg g^-1^ fresh weight) was calculated from a curve method by L-proline.

Glycine betaine was determined through the procedure explained by Grieve and Grattan [38]. In this method, 200 mg leaf sample was mashed in liquid nitrogen, then 3 mL deionized water was added to the ground mixture and placed on a mechanical shaker at 25 °C for 16 hours. Then the filtrate was extracted and diluted in 2N H_2_SO_4_ by maintaining a 1:1 ratio. The 500 mL extract was cooled for 1 hour and homogenized in 200 mL potassium iodide-iodine reagent. The above mixture was incubated at 4 °C for 16 hours then centrifuged at 10,000 rpm at 0 °C for 15 min. At the end of the centrifugation process, periodide crystals were developed which were mixed in 9 mL solution of 1,2-dichloromethane. Later, absorbance was noted for 60 min at 365 nm. Glycine betaine (mg g^-1^ FW) was noted through the standard curve method.

The article "Seed priming with growth regulators modulates production, physiology and antioxidant defense of Indian squash (Praecitrullus fistulosus) under semi-arid conditions" was retracted in 2022. Reasons: compromised peer review; a conflict of interest; concerns about the authorship.

A fresh plant tissue sample (0.5 g) was ground in 0.1 M of 2 mL potassium phosphate buffer (pH 7 with 0.1 mM EDTA) by using a mortar and pestle (precooled). Then centrifugation was started at 4 °C at 10,000 × g for 20 minutes. The liquid was stored in ice and utilized for further determination of antioxidant activities. Lipid peroxidation was determined in terms of malondialdehyde (MDA), and measurement was noted at 532 and 600 nm. Then MDA content was determined by adopting equation formulated by Heath and Packer [39]:

$$\text{MDA}\;\left(\mu \text{mol}\;{\text{g}}^{-1}\;\text{FW}\right)=\left(\left(\text{A}532–\text{A}600\right)/155,000\right)\times 106$$

Superoxide dismutase response was calculated by using the protocol of Gupta et al. [40]. According to this protocol, the supernatant was exposed, and its presence was photochemically inhibited by decreasing nitro blue tetrazolium. Then the mixture was placed for 15 minutes in a light source (15W, lamps) at 78 μmol m^-2^ s^-1^. The optical density was measured at 560 nm from the solution by using a spectrophotometer. Catalase activity was calculated by adopting the procedure as explained by Aebi [41]. Ascorbate peroxidase performance was calculated by adopting the procedure of Amako [42]. In this procedure, a reduction in absorbance was noted at 290 nm of ascorbic acid for 90 s. The oxidation (coefficient of 2.8 mM^-1^ cm^-1^) in ascorbate caused variation in absorbance which showed the ascorbate peroxidase activity.

### Statistical analysis

Experimental treatments followed the statistical planning of randomized complete randomized design (RCBD). SAS software (Version 9.1; SAS Institute, Cary, NC, USA) [43] was applied for analysis of variance (ANOVA) and correlation on all studied parameters and their means were distinguished by least significant difference test at 5% probability [44]. Graphical presentation of data was presented by working Sigma Plot software [45].

## Results

Seed germination and growth performance of Indian squash in field conditions were improved by seed priming during both years (Table 2). Significant increase in germination, germination index, and plant height and shortening in mean germination time (*P* ≤ 0.05 were observed by seed priming with ascorbic acid (AA) at 100 mg L^-1^ (Table 2). Statistically (P ≤ 0.05) higher germination percentage (39 and 47%) and germination index (57 and 58%) were recorded for seed priming with AA during 2019 and 2020, respectively compared to control treatment of the study (Table 2). Moreover, during 2019, the germination percentage for seed priming with salicylic acid (SA) at 50 mg L^-1^ was statistically at par with AA. Furthermore, seed priming with AA shortened the time taken for mean germination by 25 and 28% during 2019 and 2020, respectively. During 2019 and 2020, the mean germination time of control, distilled water and thiourea at 500 mg L^-1^ were statistically similar. Moreover, seed priming with AA significantly increased (by 23 and 22%) the plant height as compared to control during 2019 and 2020, respectively. Briefly, AA followed by SA was concluded to be more useful in improving seed germination and growth performance of Indian squash than control, thiourea at 500 mg L^-1^, hydropriming and indole acetic acid (IAA) at 100 mg L^-1^ during the study (Table 2).

The article "Seed priming with growth regulators modulates production, physiology and antioxidant defense of Indian squash (Praecitrullus fistulosus) under semi-arid conditions" was retracted in 2022. Reasons: compromised peer review; a conflict of interest; concerns about the authorship.

**Table 2:** The influence of seed priming with different growth regulators on seed germination, germination index, mean germination time, and plant height of Indian squash under field conditions.

Treatments	Germination (%)		Germination index		Mean germination time (days)		Vine length (cm)	
	2019	2020	2019	2020	2019	2020	2019	2020
**Control**	55 d	50 d	3.26 f	3.24 f	9.80 a	10.18 a	101 d	99 e
**Distill water**	65 c	65 c	4.07 d	4.07 d	10.01 a	10.08 a	109 c	107 d
**Indole acetic acid at 100 mg L** ^**-1**^	75 b	75 b	5.36 c	5.36 c	7.71 bc	7.73 bc	117 b	113 c
**Salicylic acid at 50 mg L** ^**-1**^	85 a	80 b	5.87 b	5.86 b	8.20 b	8.23 bc	127 a	122 b
**Ascorbic acid at 100 mg L** ^**-1**^	90 a	95 a	7.71 a	7.73 a	7.36 c	7.31 c	131 a	127 a
**Thiourea at 500 mg L** ^**-1**^	60 cd	55 d	3.52 e	3.51 e	9.65 a	8.92 ab	106 c	103 de
**LSD (0.05)**	8.89	8.90	0.01	0.02	0.63	1.56	4.54	4.56

Different alphabets in the column showed statistical difference (*P* ≤ 0.05) among treatments.

Temperature fluctuation in field conditions markedly decreased the production in the control treatment as compared to seed priming with growth regulators during both years of study (Table 3). However, seed priming with AA significantly enhanced vines length (120 and 116 cm) followed by SA during 2019 and 2020, respectively (Table 3). Similarly, the number of fruits per plant was 21 when AA was applied during both study years. Seed priming with AA notably increased fruit weight per plant (1124 and 1115 g) as compared to control during 2019 and 2020, respectively (Table 3). Moreover, economic yield (2415 and 2403 kg ha^-1^) was significantly (*P* ≤ 0.05) higher in the plants grown out from seed primed with AA during 2019 and 2020, respectively (Table 3). Seed priming with thiourea, distilled water, and IAA showed lower economic yield during the current study compared with SA and AA (Table 3).

The article "Seed priming with growth regulators modulates production, physiology and antioxidant defense of Indian squash (Praecitrullus fistulosus) under semi-arid conditions" was retracted in 2022. Reasons: compromised peer review; a conflict of interest; concerns about the authorship.

**Table 3:** The influence of seed priming with different growth regulators on vine length, number of fruits and fruit weight per plant and economic yield of Indian squash under field conditions.

Treatments	Vines length (cm)		Numbers of fruits per plant		Fruit weight per plant (g)		Economical yield (Mg/ha)	
	2019	2020	2019	2020	2019	2020	2019	2020
**Control**	102 e	100 e	8 d	8 c	102 e	100 e	16.3 d	16.4 c
**Distill water**	105 d	103 d	11 c	10 c	105 d	103 d	18.6 c	18.7 c
**Indole acetic acid at 100 mg L** ^**-1**^	110 c	106 c	13 c	14 b	110 c	106 c	20.6 c	20.8 b
**Salicylic acid at 50 mg L** ^**-1**^	115 b	110 b	18 b	16 b	115 b	110 b	23.2 b	23.3 b
**Ascorbic acid at 100 mg L** ^**-1**^	120 a	116 a	21 a	21 a	120 a	116 a	24.2 a	24.2 a
**Thiourea at 500 mg L** ^**-1**^	104 d	104 d	11 c	9 c	104 d	104 d	17.5 c	17.5 c
**LSD (0.05)**	1.79	1.80	2.40	2.96	1.79	1.80	2.40	2.96

Different alphabets in the column showed statistical difference (*P* ≤ 0.05) among treatments.

Photosynthesis rate was lower in the control treatment as compared to seed priming treatments. Seed priming with AA significantly enhanced the photosynthesis rate (3.84 and 3.82 μmol m^-2^ s^-1^) which was statistically at par with SA (Table 4). Similarly, protein contents (3.72 and 3.46 mg g^-1^ FW) were significantly (*P* ≤ 0.05) increased because of seed priming with AA compared to control treatment during both years of the study. Furthermore, seed priming with AA, SA and IAA alleviated the harmful effects of the heat stress (Table 4). Seed priming with AA significantly (*P* ≤ 0.05) enhanced proline content (7.99 and 7.98 μg g^-1^ FW) compared with control during each year of the study. Glycine betaine contents (252 and 250 μg g^-1^ FW) were significantly (*P* ≤ 0.05) higher in leaf tissues of plants treated with AA as compared to the control during both years of study (Table 4). It can be concluded from the results of physiological characteristics that AA and SA improved the physiological performance of Indian squash than control, thiourea, and distilled water during the study (Table 4).

**Table 4:** The influence of seed priming with different growth regulators on photosynthesis rate, protein, proline, and glycine betaine contents of Indian squash under field conditions.

Treatments	Photosynthesis rate (μmol m^-2^ s^-1^)		Protein contents (mg g^-1^ FW)		Proline (μg g^-1^ FW)		Glycine betaine (μg g^-1^ FW)	
	2019	2020	2019	2020	2019	2020	2019	2020
**Control**	3.17 d	3.15 d	3.37 d	3.11 d	6.17 e	6.16 e	240 d	238 c
**Distill water**	3.48 bc	3.45 c	3.47 cd	3.21 cd	7.17 c	7.15 c	245 bc	244 b
**Indole acetic acid at 100 mg L** ^**-1**^	3.53 bc	3.57 bc	3.54 bc	3.29 bc	7.44 bc	7.42 bc	246 b	246 b
**Salicylic acid at 50 mg L** ^**-1**^	3.68 ab	3.70 ab	3.64 ab	3.38 ab	7.75 ab	7.76 ab	247 b	247 b
**Ascorbic acid at 100 mg L** ^**-1**^	3.84 a	3.82 a	3.72 a	3.46 a	7.99 a	7.98 a	252 a	250 a
**Thiourea at 500 mg L** ^**-1**^	3.41 c	3.39 c	3.40 cd	3.17 cd	6.60 d	6.62 d	242 cd	240 c
**LSD (0.05)**	0.19	0.20	0.11	0.12	0.40	0.42	3.44	3.46

Different alphabets in the column showed statistical difference (*P* ≤ 0.05) among treatments.

The article "Seed priming with growth regulators modulates production, physiology and antioxidant defense of Indian squash (Praecitrullus fistulosus) under semi-arid conditions" was retracted in 2022. Reasons: compromised peer review; a conflict of interest; concerns about the authorship.

Seed priming with AA under field conditions increased MDA accumulation (9.13 and 9.15 μmol g^-1^ FW) during 2019 and 2020, respectively (Fig 2), while AA was statistically at par with SA. Fig 3 described that the priming with growth regulators did not affect the SOD activity during both years of study. The CAT activity (1.62 and 1.64 m Kat mg^-1^ protein) was noticeably increased in the leaf tissues by seed priming with AA during study years (Fig 4), while AA was statistically similar with SA. Fig 5 showed a non-significant improvement in APX activity in the leaf of plants grown from seeds primed with growth regulators during both years. In summary, AA and SA were useful for improving antioxidant enzymes performance in Indian squash during the study period (Figs 2 to 5).

**Fig 2:** The influence of seed priming with different growth regulators on MDA contents of Indian squash. The error bars represent ± standard error of the means. Alphabets on bar showed a significant difference (*P* ≤ 0.05) among seed priming techniques.

**Fig 3:** The influence of seed priming with different growth regulators on SOD contents of Indian squash. The error bars represent ± standard error of the means. Alphabets on bar showed a significant difference (*P* ≤ 0.05) among seed priming techniques.

**Fig 4:** The influence of seed priming with different growth regulators on CAT contents of Indian squash. The error bars represent ± standard error of the means. Alphabets on bar showed a significant difference (*P* ≤ 0.05) among seed priming techniques.

**Fig 5:** The influence of seed priming with different growth regulators on APX contents of Indian squash. The error bars represent ± standard error of the means. Alphabets on bar showed a significant difference (*P* ≤ 0.05) among seed priming techniques.

Correlation analysis between growth, yield and biochemical attributes revealed that seed germination had a strong significant (*P* ≤ 0.05) positive correlation with germination index, vine length, number of fruits per plant, fruit weight, economic yield, photosynthesis rate, proline content, glycine betaine, and MDA contents, while non-significant negative correlation was recorded with mean germination time, SOD activity, CAT activity, and APX activity (Tables 5 and 6). The economic yield had a strong significant (*P* ≤ 0.05) positive correlation with photosynthesis rate, proline content, glycine betaine, MDA contents, and CAT activity, while exhibited non-significant correlation with protein contents, SOD activity, and APX activity (Tables 5 and 6). Proline contents revealed a highly significant (*P* ≤ 0.05) positive correlation with glycine betaine, MDA contents, and CAT activity, while had non-significant correlation with SOD activity and APX activity (Tables 5 and 6).

The article "Seed priming with growth regulators modulates production, physiology and antioxidant defense of Indian squash (Praecitrullus fistulosus) under semi-arid conditions" was retracted in 2022. Reasons: compromised peer review; a conflict of interest; concerns about the authorship.

**Table 5:** *Pearson*´s correlation among different growth, yield and biochemical attributes of Indian squash during 2019.

	GER	GI	MGT	PH	VLP	NFP	FW	EY	PHR	PRC	PRO	GLB	MDA	SOD	CAT	APX
GER	---															
GI	0.92**	---														
MGT	-0.86**	-0.87**	---													
PH	0.88**	0.95**	-0.80**	---												
VLP	0.90**	0.98**	-0.83**	0.99**	---											
NFP	0.85**	0.94**	-0.73**	0.97**	0.97**	---										
FW	0.94**	0.98**	-0.87**	0.97**	0.98**	0.95**	---									
EY	0.94**	0.96**	-0.84**	0.99**	0.98**	0.95**	0.99**	---								
PHR	0.70**	0.85**	-0.62^NS^	0.93**	0.91**	0.93**	0.89**	0.88**	---							
PRC	0.03^NS^	0.30^NS^	-0.06^NS^	0.47^NS^	0.41^NS^	0.46^NS^	0.31^NS^	0.33^NS^	0.65^NS^	---						
PRO	0.79**	0.88**	-0.71**	0.95**	0.91**	0.91**	0.93**	0.93**	0.96**	0.94**	---					
GLB	0.70*	0.88**	-0.66^NS^	0.91**	0.90**	0.90**	0.89**	0.87**	0.97**	0.92**	0.96**	---				
MDA	0.75**	0.87**	-0.69^NS^	0.97**	0.94**	0.93**	0.91**	0.93**	0.96**	0.91**	0.97**	0.94**	---			
SOD	-0.02^NS^	0.28^NS^	-0.11^NS^	0.45^NS^	0.40^NS^	0.42^NS^	0.30^NS^	0.31^NS^	0.63^NS^	0.62^NS^	0.55^NS^	0.63^NS^	0.63^NS^	---		
CAT	0.64^NS^	0.80**	-0.64^NS^	0.91**	0.87**	0.87**	0.84**	0.85**	0.95**	0.72**	0.96**	0.94**	0.98**	0.74**	---	
APX	0.09^NS^	0.38^NS^	-0.20^NS^	0.55^NS^	0.49^NS^	0.51^NS^	0.40^NS^	0.41^NS^	0.71**	0.52^NS^	0.63^NS^	0.71**	0.71**	0.99**	0.81**	---

Here, Germination = GER; Germination index = GI; Mean germination time (Days) = MGT; Plant height = PH; Vines length per plant = VLP; Number of fruits per plant = NFP; Fruit weight per plant = FW; Economic yield = EY; Photosynthesis rate = PHR; Protein contents = PRC; Proline content = PRO; Glycine betaine = GLB; MDA contents = MDA; SOD activity = SOD; CAT activity = CAT; APX activity = APX. NS–non-significant;

*–significant at *P* ≤ 0.05;

**–significant at *P* ≤ 0.01.

**Table 6:** *Pearson*´s correlation among different growth, yield, and biochemical attributes of Indian squash during 2020.

	GER	GI	MGT	PH	VLP	NFP	FW	EY	PHR	PRC	PRO	GLB	MDA	SOD	CAT	APX
GER	---															
GI	0.96**	---														
MGT	-0.75**	-0.71**	---													
PH	0.98**	0.95**	-0.73**	---												
VLP	0.95**	0.96**	-0.74**	0.97**	---											
NFP	0.98**	0.95**	-0.77**	0.97**	0.96**	---										
FW	0.96**	0.98**	-0.74**	0.97**	0.96**	0.95**	---									
EY	0.95**	0.96**	-0.70*	0.98**	0.95**	0.94**	0.99**	---								
PHR	0.96**	0.86**	-0.75**	0.95**	0.92**	0.94**	0.90**	0.90**	---							
PRC	0.03^NS^	0.30^NS^	-0.06^NS^	0.47^NS^	0.41^NS^	0.46^NS^	0.31^NS^	0.33^NS^	0.65^NS^	---						
PRO	0.97**	0.88**	-0.71**	0.96**	0.90**	0.93**	0.93**	0.93**	0.98**	0.96**	---					
GLB	0.98**	0.89**	-0.71**	0.94**	0.90**	0.94**	0.91**	0.90**	0.97**	0.97**	0.98**	---				
MDA	0.96**	0.87**	-0.74**	0.97**	0.91**	0.95**	0.92**	0.93**	0.98**	0.99**	0.98**	0.97**	---			
SOD	-0.08^NS^	0.23^NS^	-0.45^NS^	0.42^NS^	0.37^NS^	0.48^NS^	0.25^NS^	0.27^NS^	0.60^NS^	0.63^NS^	0.51^NS^	0.57^NS^	0.58^NS^	---		
CAT	0.53^NS^	0.80**	-0.73**	0.92**	0.86**	0.92**	0.84**	0.86**	0.97**	0.98**	0.95**	0.95**	0.98**	0.72**	---	
APX	0.57^NS^	0.34^NS^	-0.50^NS^	0.52^NS^	0.46^NS^	0.57^NS^	0.36^NS^	0.37^NS^	0.68^NS^	0.71^NS^	0.60^NS^	0.66^NS^	0.66^NS^	0.99**	0.79**	---

Here, Germination = GER; Germination index = GI; Mean germination time (Days) = MGT; Plant height = PH; Vines length per plant = VLP; Number of fruits per plant = NFP; Fruit weight per plant = FW; Economic yield = EY; Photosynthesis rate = PHR; Protein contents = PRC; Proline content = PRO; Glycine betaine = GLB; MDA contents = MDA; SOD activity = SOD; CAT activity = CAT; APX activity = APX. NS–non-significant;

*–significant at *P* ≤ 0.05;

**–significant at *P* ≤ 0.01.

The article "Seed priming with growth regulators modulates production, physiology and antioxidant defense of Indian squash (Praecitrullus fistulosus) under semi-arid conditions" was retracted in 2022. Reasons: compromised peer review; a conflict of interest; concerns about the authorship.

## Discussion

Indian squash is a sensitive crop to extreme environmental fluctuation that can be improved by seed priming. The present study confirmed our hypothesis and significant improvement in seed germination, production, physiology, and antioxidant enzymes characteristics of were recorded through priming with ascorbic acid and salicylic acid under field conditions (Tables 2 to 4 and Figs 2 to 5). Moreover, the current experiments revealed that ascorbic acid and salicylic acid alleviated the harmful impact of temperature (Figs 2 to 5 and Tables 2 to 4). Seed priming with ascorbic acid and salicylic acid resulted in improved seed germination characteristics during both years (Table 2). This improvement in germination characteristics [23] might be possible due to improvement in plant defense system, i.e., MDA contents that have a positive correlation with seed germination (Tables 5 and 6). Moreover, our study supported the findings of Qamar et al. [23] who reported that priming with ascorbic acid and salicylic acid brings uniformity and synchronization in germination % and shortening in mean germination time are important signs for healthy crop establishment. However, improvement in germination characteristics by ascorbic acid and salicylic acid seed priming compared with other seed priming treatments might be due to the involvement of these growth regulators in metabolic reactions of hormones and antioxidant enzymes system that led to improved biochemical processes in seed germination such as hydrolysis, enzymes energizing and dormancy diminishing, which is necessary to initiate germination process [21]. Taller plants were recorded for seeds primes with ascorbic acid and salicylic acid (Table 2) during both years of study. The possible justification for this significant improvement in plant height is the enhancement in plant metabolism through protecting cells from reactive oxygen species (Figs 2 to 5 and Tables 5 and 6) as production of free radicals increases during the environmental fluctuation [46, 47]. In the control treatment, higher accumulation of reactive oxygen species probably restricted cell multiplication and expansion that leads to shorter plant height, while growth regulators improved the antioxidative potential of cells [23, 48].

The article "Seed priming with growth regulators modulates production, physiology and antioxidant defense of Indian squash (Praecitrullus fistulosus) under semi-arid conditions" was retracted in 2022. Reasons: compromised peer review; a conflict of interest; concerns about the authorship.

The improvement in vine length, fruits number, weight, and economic yield due to seed priming with ascorbic acid and salicylic acid in the present study (Table 3) might be due to improvement in early emergence on account of metabolic and biochemical processes occurring during controlled hydration. Controlled hydration promoted radicle to protrusion [49]; thus, supported the production traits depicted in correlation analysis (Tables 5 and 6). Such significant (P ≤ 0.05) modifications were predicted due to swift stimulation of physiological processes [50] in germination than non-primed seeds. As a result of higher cell division and cell elongation by keeping the hormonal balance in the plant tissues, cell multiplication was speeded up by increasing the internal level of other regulators of plant growth [17]. Our results supported the conclusions of Guo et al. [51] who reported significant improvement in morphological development and biomass accumulation in the root system due to the application of growth regulators. Ascorbic acid and salicylic acid are indirectly involved in flower production due to their connection with growth hormones production [52] that encourages flowering [53] and limits senescence [54].

Improvement in photosynthesis rate was recorded with ascorbic acid and salicylic acid priming in the current study (Table 4). Many investigators reported that improvement in photosynthesis rate could be possible due to large surface area of leaves which had a significant correlation with developmental traits (Tables 5 and 6). Our results supported the conclusion of Haung et al. [55] and Qamar et al. [23] who reported that growth regulators might increase the concentration of carotenoids which leads to improvement in photosynthesis rate. An increase in protein content due to seed priming with ascorbic acid (Table 4) is in harmony with earlier findings [23, 56]. A strong positive correlation of protein content with antioxidants further strengthened it (Tables 5 and 6). In this regard, higher accumulation of proline in plant tissues for carrying out osmotic adjustment played a significant role as an osmotic regulator; thus, reducing high-temperature stress [57].

The article "Seed priming with growth regulators modulates production, physiology and antioxidant defense of Indian squash (Praecitrullus fistulosus) under semi-arid conditions" was retracted in 2022. Reasons: compromised peer review; a conflict of interest; concerns about the authorship.

Higher production of MDA contents by ascorbic acid and salicylic acid treatments restricted the membrane fluidity and leakage from cells and membrane, moreover protected membrane proteins, enzymes, and ion channels [58]. The present study showed that seed priming with ascorbic acid and salicylic acid increased SOD activity by restricting the increase of H_2_O_2_; thus, performed as a direct ROS scavenger (Figs 3 and 4) [59]. Results of both years depicted that seed priming with ascorbic acid at 100 mg L^-1^ and salicylic acid at 50 mg L^-1^ improved SOD and CAT activity in leaves by limiting the accumulation of H_2_O_2_ in intercellular spaces (Figs 3 and 4) [59, 60]. Our study showed a non-significant effect of seed priming on ascorbate peroxidase concentration, while findings of Zhang [61] demonstrated a higher concentration of ascorbate peroxidase that is an important component of glutathione ascorbate cycle and is directly involved in detoxification of cells under high-temperature stress. The other cause may be an improvement in gas exchange processes that promoted stomatal opening and encouraged lowering canopy temperature and higher CO_2_ exchange [62]. In the current study, hydropriming doesn’t show significant results than growth regulators; however, it was better than non-primed seed which could be possible due to enhanced rehydrating seeds [63].

## Conclusion

Food security is the main challenge in agricultural crop production under environmental fluctuation during the present era. The results of the current study revealed that seed priming with ascorbic acid at 100 mg L^-1^ and salicylic acid at 50 mg L^-1^ proved effective in enhancing seed germination, growth characteristics and yield attributes of Indian squash because of improved plant physiological processes and antioxidant enzymes properties which altogether mitigated the adverse impacts of heat stress under field conditions. Seed priming with ascorbic acid and salicylic acid can be used to impart heat-tolerance to Indian squash under semi-arid climatic conditions.
